This article has been retracted.

# Effects of Adipose Plasma Transfusion Compared with Normal Plasma Transfusion on Adverse Transfusion Reactions, Important Functional Indicators, and Clinical Safety in Patients with Parenteral Nutrition: Based on a Retrospective Cohort Study

**DOI:** 10.1155/2022/6089771

**Published:** 2022-08-12

**Authors:** Chunhong Gong, Xingxing Qin, Hongxia Chen, Xing Wu, Juan Wu, HuaMin Li, Wei Wang

**Affiliations:** ^1^Xianning Central Hospital (The First Affiliated Hospital of Hubei University of Science and Technology) Blood Transfusion Department, Xianning, Hubei 437100, China; ^2^Xianning Central Hospital (The First Affiliated Hospital of Hubei University of Science and Technology) Gastrointestinal Surgery, Xianning, Hubei 437100, China; ^3^Xianning Central Hospital (The First Affiliated Hospital of Hubei University of Science and Technology) Gastroenterology Department, Xianning, Hubei 437100, China; ^4^Xianning Central Blood Bank, Xianning, Hubei 437100, China

## Abstract

**Objective:**

Based on a retrospective cohort study, the study aims to investigate the effects of adipose plasma transfusion compared with normal plasma transfusion on adverse transfusion reactions, important functional indicators, and clinical safety in patients with parenteral nutrition (PN).

**Methods:**

One hundred and twenty inpatients who needed PN and plasma transfusion in Xianning Central Hospital from September 1, 2021, to March 31, 2022, were enrolled as the actual application verification cases. All the patients in the group noticed the informed consent form, and the normal plasma transfusion was set as the control group (*n* = 40), and the fat plasma transfusion was set as the study group. Mild adipose plasma transfusion was adopted in study group ① and moderate adipose plasma transfusion was used in study group ②, 40 cases in each group. The blood routine tests, blood lipids, blood coagulation, liver function tests, and the incidence of adverse reactions of blood transfusion were compared.

**Results:**

The comparison results of platelet count, red blood cell count, hemoglobin, and hematocrit among the three groups are as follows: study group ②> study group ①> control group (*P* < 0.05).The levels of blood lipids in the three groups, triglyceride, total cholesterol, high density lipoprotein, and low density lipoprotein were compared in group ②>group ①>control group (*P* < 0.05).The liver function tests indexes of the three groups were compared: ALT, AST, LDH: study ②<study ①<control group; ALP: study ②>study ①>control group. Regarding the incidence of adverse transfusion reactions, the incidence of adverse transfusion reactions in the study group was lower than in the control group (*P* < 0.05).

**Conclusion:**

Compared with normal plasma transfusion, the inpatients who need PN and plasma transfusion can effectively use the scrapped mild and moderate fatty plasma and reduce the plasma scrap rate. In the meantime, it has little effect on the function of the important indexes of the patients, and the incidence of adverse reactions of blood transfusion is low and the safety is high. Infusion of adipose plasma can also improve the effective individual and rational utilization of blood products. Trial registration: This trial is registered with chiCTR220005918.

## 1. Introduction

The World Health Organization (WHO) proposed that when the blood donation rate of a country reaches 10‰∼30‰, it can basically meet the needs of some clinical blood use. After years of efforts by the government and blood collection and supply institutions, the rate of unpaid blood donation is gradually increasing. The National Commission of Health and Health reported that China's blood donation rate in 2017 was about 11 per thousand, reaching the lower level advocated by WHO [1]. However, on the one hand, with the intensification of social aging, the number of new blood donors is less than that of voluntary blood donors of the right age, and second, blood donation is also greatly affected by force majeure. For example, during the COVID-19 epidemic, the number of people donating blood decreased seriously, which became a national problem. On the other hand, with the continuous improvement of medical technology in our country, the amount of blood is increasing year by year and the situation of tight blood supply still exists [2]. In order to deal with the blood supply gap, we need to grasp with both hands. On the one hand, blood collection and supply institutions should strengthen recruitment and publicity and correctly guide blood donation; on the other hand, technical innovation should be carried out to reduce the scrapping rate of blood products of noncommunicable testing indicators [3].

With the development of economy and society, people's living conditions are getting better, and the pace of life is getting faster: bad lifestyles such as high-fat diet, night shift, and sitting for a long time make many office workers in a “sub-healthy state” [4]. Therefore, the incidence of hyperlipidemia is increasing day by day. Data from epidemiological surveys show that the prevalence of hyperlipidemia in people aged 20 to 60 in China is about 30% to 50% [5]. Among the reasons for the scrapping of noninfectious testing indicators, according to the academic reports of local blood stations, the scrapped proportion of fat plasma is the highest and the proportion of unpaid blood donation due to excessive fat content is on the rise [6]. The scrapping of fat plasma not only consumes manpower and material resources but also wastes precious blood resources. There are two aspects of clinical concern about the use of adipose plasma, on the one hand, whether the quality of adipose plasma is consistent with that of chylous plasma, and on the other hand, whether adipose plasma will cause adverse reactions of blood transfusion [7]. Many previous studies have reported that nonhemolytic fever and allergic reactions are the most common causes of adverse transfusion reactions, but these adverse transfusion reactions are not directly related to chylous particles (CM) [8]. Related literature reported that the removal of chylous particles in adipose blood samples will not affect the detection results of transfusion-related infectious disease markers and the quality meets the national quality standards [9].

In order to avoid the waste of blood, most scholars are studying how to control the production of fat plasma from the source of blood collection, such as strengthening the publicity of unpaid blood donation knowledge, popularizing the physiological knowledge of unpaid blood donation, strict physical examination consultation, and other methods [10]. However, under the condition that blood resources are still so precious, it is particularly important for clinical blood transfusion department to control clinical scientific and rational use of blood, save blood, and protect limited blood resources through fine management of clinical blood use [11]. Scientific and rational blood transfusion should proceed from the actual situation of patients and formulate individualized blood transfusion plan. PN refers to the intravenous administration of appropriate amount of protein (amino acids), fats, carbohydrates, electrolytes, vitamins, and trace elements to patients who are unable to absorb nutrients through the gastrointestinal tract or who cannot meet their own metabolic needs, so as to inhibit catabolism, promote the synthesis of metabolic diseases, maintain the function of structural proteins, and achieve the purpose of nutritional therapy. PN has been widely adopted in clinic, but there are few reports about the application of adipose plasma. We intend to study the rationality of using adipose plasma in clinic to explore whether the blood use can be reasonable and economical through the rational use of mild and moderate adipose plasma in the case of patients who need plasma transfusion because of their condition and fat transfusion through PN [12]. The purpose of this study was to explore the possibility of rational use of mild and moderate adipose plasma by comparing the adverse reaction monitoring, blood routine tests, blood lipid, thromboelastogram, and liver function tests indexes of normal plasma + PN, mild adipose plasma + PN, and moderate adipose plasma + PN. The goal of this project is to effectively utilize the scrapped mild and moderate fatty plasma, reduce the plasma scrapping rate, alleviate the current shortage of blood resources, and enhance the effective individual and rational utilization of blood products. It has a very important economic value and social value.

## 2. Patients and Methods

### 2.1. General Information

One hundred and twenty inpatients who needed PN and plasma transfusion in Xianning Central Hospital from September 1, 2021, to March 31, 2022, were enrolled as the actual application verification cases. All the patients in the group noticed the informed consent form, and the normal plasma transfusion was set as the control group (*n* = 40), and the fat plasma transfusion was set as the study group. Mild adipose plasma transfusion was adopted in study group ① and moderate adipose plasma transfusion was used in study group ②, 40 cases in each group. In the control group, the age was 20–75 years old, with an average of (42.54 ± 3.66) years, including 14 males and 26 females. In group ①, the age ranged from 20 to 75 years old, with an average of (42.96 ± 3.53) years, including 17 males and 23 females. In group ②, the age ranged from 20 to 75 years old, with an average of (43.55 ± 3.78) years, including 18 males and 22 females. There was no no statistical significance in the general data.

Inclusion criteria were as follows: (1) 20–75 years old; (2) 70 males and 50 females; (3) upper gastrointestinal obstruction, colonic obstruction, colorectal obstruction, and nonhyperlipidemic pancreatitis in gastroenterology; (4) preoperative or postoperative patients with gastric cancer, colon tumor, rectal tumor, liver cancer, pancreatic cancer, cholangiocarcinoma, hepatolithiasis, etc.; (5) patients with malnutrition such as plasma transfusion and PN; (6) the cardiopulmonary function is normal; and (7) know the scheme, points for attention and possible complications of this study and sign the informed consent form with full informed consent.

Exclusion criteria were as follows: (1) previous history of blood transfusion; (2) hematological diseases; (3) familial and hereditary hyperlipidemia; (4) severe hepatorenal dysfunction or immune system diseases; (5) allergy to nutrients or infusion taboos; (6) history of using drugs that affect the test; and (7) thrombus.

### 2.2. Treatment Methods

First, we educate the patient bed-care physicians and nurses on the matters needing attention and distribute the “adverse reaction questionnaire” and the operation manual [13]. Clinical medical staff should pay attention to the implementation of health education for patients and give timely and effective psychological nursing intervention. For patients with impatience, they should tell patients not to be impatient and to maintain a stable state of mind to accept all kinds of treatment and nursing. And inform patients of some clinical symptoms that may occur in the process of drug infusion, such as nausea and vomiting, appease patients not to worry too much, and teach patients to timely and correctly describe self-conscious symptoms. In order to be able to find the existence of the problem at the first time, we take effective measures to intervene in time and explain to the patients and their families the importance, purpose, significance, and implementation methods of infusion of plasma and fat emulsion injection, so that they can have a psychological preparation in advance and constantly improve their awareness, which is an important factor to ensure active cooperation and achieve ideal therapeutic results. Medical staff should timely find the abnormal situation of the patient and inform the doctor in time to deal with it.

Blood transfusion department incubates plasma in accordance with standard operating procedures. Obvious bubbles, flocs, or coarse particles in plasma are not allowed to be emitted. Plasma was infused within 30 minutes after clinical delivery. Plasma was infused first, and the infusion process was operated according to the standard required by the Technical Specification for Clinical Blood Transfusion [14]. The speed of intravenous drip is slower in the first 15 minutes, and the general speed is 5∼10 ml/min, about 750∼150 drops/min. The first infusion dose was 10∼15 ml/kg and the maintenance dose were 5∼10 ml/kg.

### 2.3. Observation Indicators

#### 2.3.1. Laboratory Indicators

Blood routine tests, blood lipids, blood coagulation, and liver function tests were conducted. The venous blood of the patient was drawn for 3 ml and an anticoagulant was added to the blood sample. The blood routine test, blood lipids, and liver function test indexes in blood samples were detected by an automatic blood biochemical analyzer and matching reagents. The method of coagulation function test is as follows: the venous blood of the patient is collected for 2 ml, and the blood sample is centrifuged for 15 min to separate the plasma. The blood coagulation indexes were detected by an automatic blood coagulation analyzer. Coagulation function: plasma fibrinogen, thrombin time, activated partial thromboplastin time, prothrombin time. blood routine tests (platelet count, red blood cell count, hemoglobin, and hematocrit). Four items of blood lipids: triglyceride, cholesterol, low density lipoprotein, high density lipoprotein. Liver function tests: ALT, AST, ALP, LDH.

### 2.4. Adverse Reactions to Blood Transfusion

The adverse reaction monitoring cards of the three groups were collected, and the adverse reaction rate was calculated according to the number of adverse reactions assigned by the percentage of total blood transfusions.

### 2.5. Statistical Analysis

Using SPSS 21.0 statistical software, before statistical analysis, the measurement data were examined by normal distribution and variance homogeneity analysis to meet the requirements of normal distribution or approximate normal distribution, presented as $\bar{x}$ ± *s*, and repeated measurement data were analyzed by repeated measurement analysis of variance. The *T* test was adopted to compare, taken *n* (%) as an example to represent counting data, and performed *χ*^2^ test, *P* < 0.05 indicates that the difference is statistically significant.

## 3. Results

### 3.1. Comparison of Blood Routine Tests Indexes

The comparison results of platelet count, red blood cell count, hemoglobin, and hematocrit among the three groups are as follows: study group ②> study group ①> control group (*P* < 0.05). All the data results are indicated in Table 1.

### 3.2. Comparison of Blood Lipid Levels

In terms of blood coagulation indexes and plasma fibrinogen among the three groups, study group②<study group①<control group. The comparison of thrombin time, activated partial thromboplastin time, and prothrombin time among the three groups was as follows: study group ②>study group ①>control group (*P* < 0.05). All the data results are indicated in Table 2.

### 3.3. Comparison of Liver Function Test Indexes

With regard to liver function tests indexes among the three groups, ALT, AST, and LDH, study group②<study group①<control group, compared with the three groups of ALP, study group②>study group①>control group (*P* < 0.05). All the data results are indicated in Figure 1.

### 3.4. Comparison of the Incidence of Adverse Reactions to Blood Transfusion

Regarding the incidence of adverse transfusion reactions, the incidence of adverse transfusion reactions in the study group was lower compared to that of the control group (*P* < 0.05). All the data results are indicated in Figure 2.

## 4. Discussion

Nutritional support includes enteral nutrition directly into the gastrointestinal tract (EN) and intravenous parenteral nutrition (PN) [15]. For critically ill patients, enteral nutrition can play a role in the following ways. On the one hand, enteral nutrition helps to maintain the mechanical barrier of intestinal mucosa by maintaining the normal structure, intercellular connection, and villus height of intestinal mucosa, which is of great significance to the nursing quality of patients after operation and the management of daytime ward [16, 17]. There are more than 70% of lymphoid tissues in the gastrointestinal tract. Therefore, the gastrointestinal tract acts not only as a digestive organ but also as a major immune organ. When enteral nutrition is initiated, gastric acid, pepsin, and IgA are secreted, which help maintain the balance of biological, immune, and chemical barriers of the mucosa and maintain the growth of intestinal flora [18]. On the other hand, enteral nutrition can effectively restore the ability to stimulate blood lymphocytes, promote the renewal of intestinal cells, and maintain intestinal function. Enteral nutrition is a method of providing nutrition directly to the stomach and small intestine through the mouth, digestive tract, or artificial cavity. Enteral nutrition cannot be adopted for intestinal failure or severe inflammation without normal function, or for intestines that do not have defecation after surgery or early multiple trauma. In addition, severe burns or multiple injuries may not apply [19].

PN is subassigned into total parenteral nutrition (TPN) and supplementary parenteral nutrition (SPN) [20]. TPN refers to when patients with gastrointestinal dysfunction or failure, cannot be enteral nutrition or do not allow enteral nutrition, through the central vein, or peripheral intravenous infusion of necessary nutrients to meet the comprehensive metabolic needs. This is the only way of nutritional support. SPN is suitable for the stage of complete insufficiency of enteral nutrition or the transition from total PN to enteral nutrition. In the same time of enteral nutrition, essential nutrients should be supplemented from vein. Enteral nutrition helps to maximize gastrointestinal function.

Enteral nutrition can maintain intestinal mucosal absorption function and stimulate the recovery of gastrointestinal peristaltic function, but some patients have poor tolerance in the early stage after operation [21]. In addition, the use of enteral nutrition alone may be seriously related to malnutrition and there may be some restrictions on the use of severe patients. Naomi et al. reported that patients received about 59% of their daily calories only through enteral nutrition in the first 12 days in the intensive care unit [22]. In many guidelines and larger randomized trials, it is difficult for patients to fully achieve their goals by receiving enteral nutrition alone, and it takes a long time to achieve their goals [23]. On the contrary, PN can rapidly enhance the nutritional status of critically ill patients, and the absorption of nutrients cannot be affected by intestinal mucosal function, but long-term PN can lead to intestinal barrier dysfunction, intestinal flora imbalance and liver function tests damage [24]. Moreover, fewer patients with vomiting and diarrhea caused by PN may feel more comfortable than enteral nutrition alone [25]. Because of its advantages, PN has been used 35% to 70% clinically. Therefore, this study believes that perioperative administration of EN before operation, early use of PN combined with EN and then gradual transition to EN regimen can further enhance the nutritional status of patients than simple EN or PN regimen, more reasonable and promote rapid recovery [26].

Fatty blood is also called chylous blood. After the fat ingested by the human body is digested and absorbed in the small intestine, it becomes tiny chylous particles into the blood [27]. When chylous particles are numerous to a certain extent, the serum changes from a clear and transparent yellowish liquid to a milky sticky liquid. Medically known as chylous blood, it means that there is a high amount of fat in the blood. There are many kinds of lipids, among which cholesterol and triglyceride are more well-known [28]. Cholesterol is the most abundant steroid compound in the body. It is not only a component of cell biofilm and lipoprotein but can also synthesize cholic acid and vitamin Dand is a precursor of steroid hormones; so; for most tissues, the supply of cholesterol and the maintenance of metabolic balance are very important [29]. The sources of sterols in the human body include synthesis in the body and intake from food, but plant-based foods do not contain cholesterol, but plant sterols, which are not easily absorbed by the human body [30]. Excessive intake will inhibit the absorption of cholesterol. Triglycerides are the most abundant lipids in the human body and most tissues can use the products decomposed by triglycerides to provide calories [31]. Chylous blood lipids are important energy sources for the human body, just as gasoline is an important source of energy for automobiles. Lipids are carried to all parts of the body through lipoproteins to provide energy needs or storage [32]. Fatty blood is related to many factors, including age, sex, physique, health status, and pre-donation diet of blood donors, among which pre-diet is a more common factor. For example, eating a large amount of high-fat food within 5-6 hours before blood donation led to a significant increase in blood lipid content. However, this kind of blood cannot be donated to others, donors also need to pay special attention to whether there is dyslipidemia, such as hyperlipidemia, the proportion of chylous blood among some blood donors is as high as 1% [33].

With the change of people's lifestyle and diet and blood donation after meal, more chylous blood is collected from the blood station [34]. The quality standard of chylous plasma is established in the national standard of the people's Republic of China GB 18469Mel 2012 “quality requirements of whole blood and component blood.” The blood station also selects chylous blood according to this standard. In order to make good use of precious blood, some scholars have discussed the method of low temperature inverted centrifugation to remove chylous particles in plasma and achieved good results [35]. Some scholars have investigated the distribution of the incidence of chylous blood in different blood donors and instructed blood institutions to take corresponding countermeasures when recruiting blood donors, such as asking blood donors seriously and in detail about their diet before blood donation. One should do a good job in pre-recruitment publicity and notice before blood donation, so that blood donors can reasonably control their diet before blood donation [36].

At present, the problem of insufficient blood supply in China is becoming more serious [37]. In order to make rational use of chylous plasma, clinical blood transfusion department through fine management of clinical blood use, it is particularly important to control clinical scientific and rational use of blood, save blood, and protect limited blood resources [38]. Scientific and rational blood transfusion should proceed from the actual situation of patients and formulate individualized blood transfusion plan. Fresh frozen plasma is suitable for bleeding caused by lack of coagulation factors and diseases requiring blood volume or plasma protein supplementation, such as severe trauma, surgical bleeding, massive blood transfusion, plasma exchange, cardiopulmonary bypass, disseminated intravascular coagulation, liver cirrhosis, hypoproteinemia, neonatal hemolysis, and thrombotic thrombocytopenic purpura. Chylous particles are the largest lipoprotein particles in human plasma, mainly derived from food fat, synthesized by intestinal mucosal cells, and are the main form of dietary triglyceride transport in the body. The reassembled triglyceride was combined with apolipoprotein in intestinal mucosal cells to synthesize chylous particles [39].

Chylous particles only appear in the blood after meals, and about maintain 30 min is rapidly degraded into triacylglycerol and chylous microparticle residues by lipoprotein lipase in muscles and adipose tissues [40]. If the clearance of chylous particles in blood is hindered due to genetic factors or the lack of lipoprotein lipase or some kind of apolipoprotein in the body, the clearance of chylous particles in blood is hindered, resulting in a significant increase in serum triacylglycerol, which is chylous in appearance, so it is usually called chylous blood. With the improvement of people's living standards, there is a large proportion of chylous blood among unpaid blood donors, and chylous concentration is not one of the primary screening items for blood donation, so the chylous blood collected from different CI has also increased year by year. There are two aspects of clinical concern about the use of chylous plasma. On the one hand, whether the quality of chylous plasma is different from that of nonchylous plasma, and on the other hand, whether chylous plasma will cause adverse reactions of blood transfusion. Previous studies have reported that the causes of adverse transfusion reactions can be assigned into hemolytic transfusion reactions and nonhemolytic transfusion reactions, of which nonhemolytic fever reactions and allergic reactions are the most common, but these adverse transfusion reactions are not directly related to chylous particles [41].

Combined with the results of this study, the blood routine test indexes of the three groups were compared, platelet count, red blood cell count, hemoglobin, and hematocrit were compared among the three groups: study group ②>study group ①> control group (*P* < 0.05). The levels of blood lipids in the three groups, triglyceride, total cholesterol, high density lipoprotein, and low density lipoprotein were compared in group ②>group ①>control group (*P* < 0.05). Comparison of blood coagulation indexes and plasma fibrinogen among the three groups, study group ②<study group ①<control group. The comparison of thrombin time, activated partial thromboplastin time, and prothrombin time among the three groups was as follows: study group ②> study group ①>control group (*P* < 0.05). In terms of liver function test indexes among the three groups, ALT, AST, and LDH, study group ②<study group ①<control group. Compared with the three groups of ALP, study group ②>study group ①>control group (*P* < 0.05). Regarding the incidence of adverse transfusion reactions, the incidence of adverse transfusion reactions in the study group was lower compared to the control group (*P* < 0.05). The analysis shows that mild to moderate adipose plasma transfusion in patients with PN will not increase the rate of adverse reactions to blood transfusion; it can also effectively make use of scrapped mild and moderate adipose plasma to alleviate the current shortage of blood resources; mild to moderate adipose plasma transfusion can achieve the desired therapeutic effect of plasma transfusion [42]. This study still has some shortcomings. First, the quality of this study is limited due to the small sample size we included in the study. Second, this research is a single-center study and our findings are subject to some degree of bias. Therefore, our results may differ from those of large-scale multicenter studies from other academic institutes. This research is still clinically significant and further in-depth investigations will be carried out in the future.

In summary, in-patients who need PN and plasma transfusion, compared with normal plasma transfusion, transfusion of fatty plasma can effectively use the scrapped mild and moderate fatty plasma and reduce the plasma scrapping rate to alleviate the current shortage of blood resources, meanwhile, it has little effect on the function of important indicators of patients, and the incidence of adverse reactions of blood transfusion is low and safe. Infusion of adipose plasma can also enhance the effective individual and rational utilization of blood products.

## Figures and Tables

**Figure 1:** Comparison of liver function indexes among three groups.

**Figure 2:** Comparison of incidence of transfusion adverse reactions among three groups.

**Table 1:** Comparison of blood routine tests indexes ($\bar{x}$ ± *s*).

Group	*N*	Platelet count (x10^9^)	Red blood cell count (x10^9^)	Hemoglobin (x10^9^)	Hematocrit (%)
C Group	40	45.55 ± 1.45	2.18 ± 0.53	60.95 ± 9.93	0.19 ± 0.04
Study group ①	40	47.53 ± 1.35	3.41 ± 0.05	67.95 ± 4.12	0.23 ± 0.04
Study group ②	40	48.52 ± 1.24	3.64 ± 0.04	68.92 ± 4.56	0.28 ± 0.05
*F*		50.237	259.466	16.639	42.807
*P*		<0.01	<0.01	<0.01	<0.01

**Table 2:** Comparison of blood coagulation indexes ($\bar{x}$ ± *s*).

Group	*N*	Plasma fibrinogen (g/L)	Thrombin time (s)	Activated partial thromboplastin time (s)	Prothrombin time (s)
C Group	40	3.59 ± 0.41	15.48 ± 1.43	26.53 ± 5.64	12.48 ± 3.56
Study group ①	40	2.85 ± 0.22	28.93 ± 3.53	34.66 ± 4.64	19.49 ± 4.33
Study group ②	40	2.34 ± 0.33	34.59 ± 4.55	39.81 ± 4.15	22.49 ± 2.45
*F*		145.679	328.405	76.239	84.617
*P*		<0.01	<0.01	<0.01	<0.01

## Data Availability

The datasets used and analyzed during the current study are available from the corresponding author upon reasonable request.
